The article "Ultrasonic Imaging of Cardiovascular Disease Based on Image Processor Analysis of Hard Plaque Characteristics" was retracted in 2023. Reasons: signs of a paper mill; compromised peer review; unreliable results or conclusions.

# Ultrasonic Imaging of Cardiovascular Disease Based on Image Processor Analysis of Hard Plaque Characteristics

**DOI:** 10.1155/2022/4304524

**Published:** 2022-10-13

**Authors:** Chunxia Wang, Yufeng Ren, Jing Li

**Affiliations:** ^1^Department of Ultrasound, Liaocheng People's Hospital, Liaocheng, 252000 Shandong, China; ^2^Department of Ultrasound, Dongchangfu Hospital of Traditional Chinese Medicine, Liaocheng, 252000 Shandong, China

## Abstract

Cardiovascular disease detection and analysis using ultrasonic imaging expels errors in manual clinical trials with precise outcomes. It requires a combination of smart computing systems and intelligent image processors. The disease characteristics are analyzed based on the configuration and precise tuning of the processing device. In this article, a characteristic extraction technique (CET) using knowledge learning (KL) is introduced to improve the analysis precision. The proposed method requires optimal selection of disease features and trained similar datasets for improving the characteristic extraction. The disease attributes and accuracy are identified using the standard knowledge update. The image and data features are segmented using the variable processor configuration to prevent false rates. The false rates due to unidentifiable plaque characteristics result in weak knowledge updates. Therefore, the segmentation and data extraction are unanimously performed to prevent feature misleads. The knowledge base is updated using the extracted and identified plaque characteristics for consecutive image analysis. The processor configurations are manageable using the updated knowledge and characteristics to improve precision. The proposed method is verified using precision, characteristic update, training rate, extraction ratio, and time factor.

## 1. Introduction

Cardiovascular disease (CVD) affects the heart due to damage to blood vessels. CVD mainly occurs due to an unhealthy diet and large consumption of tobacco. CVD detection and prediction are complicated tasks to perform in healthcare centers. Ultrasonic imaging or sonography is mainly used for CVD detection [1]. Ultrasonic imaging uses high-frequency sound waves to find a detailed view of the body. Sonograph provides an actual view of the inside of the body via images [2]. Ultrasonic imaging is also used to capture the movements of internal organs that provide an optimal set of data for various processes in healthcare centers [3]. The ultrasonic image analysis process produces a feasible dataset for the CVD diagnosis process. The ultrasonic image analysis process reduces or eliminates the large volume of information and unnecessary information presented in an image. Various algorithms and techniques are used here to provide the information required for the diagnosis process [4]. The analysis process plays a significant role in improving the accuracy [4] and performance in providing emergency services for CVD patients. The ultrasonic image analysis process reduces the error rate and latency rate in the identification process, enhancing the system's feasibility [5].

Cardiovascular disease (CVD) contains various symptoms such as high-risk plaque characteristics (HRPC) and artery disease. HRPC is also associated with CVD, which increases the risk rate for patients [6]. Various methods and techniques are used in CVD's plaque characteristic analysis process. The grey-scale median (GSM) method is commonly used for plaque identification. GSM used logistics regression analysis to fetch important data related to plaque [7]. The prognostic implication method is also used in the HRPC analysis process, identifying the plaque rate in CVD [8]. The prognostic method identifies the plaque vulnerability rate and produces an optimal dataset for the CVD detection and diagnosis process. Computer tomography angiography (CTA) is one of the most commonly used for the analysis process. CTA finds the HRPC rate in CVD and provides the necessary data for the diagnosis process. CTA reduces the error rate and false identification rate in the HRPC analysis process [9, 10].

Cardiovascular disease (CVD) detection is a complicated task in every healthcare center. CVD detection requires an accurate set of data for the detection process. CVD detection is vital in providing emergency services for patients [11]. Intelligent image processors and processing techniques are mainly used for CVD detection. Artificial intelligence- (AI-) based methods are commonly used for detection. Deep reinforcement learning (DRL) algorithm is used in the CVD detection process [12]. The feature extraction method is used in DRL that identifies the essential features and patterns that are presented in an image. DRL reduces the cost and time-consuming rate in the computation process [13]. NN identifies the actual cause of CVD and finds the exact location of CVD, reducing the latency rate in providing the diagnosis process for the patients. A big data-based CVD detection process is also used here that identifies the important set of images from a large amount of data [14, 15].

## 2. Related Works

Gago et al. [16] proposed a new framework for atherosclerotic plaque detection. The semantic segmentation model is used here to determine the carotid intima-media region that is presented in an artery. A Bayesian optimization process is also used here to improve the thickness rate of the intima-media region and provide an optimal dataset for the plaque detection process.

Yang et al. [17] introduced an automatic plaque characterization method for coronary atherosclerotic plaques. A support vector machine classifier is used here to classify the data necessary for the detection process. Important features are first identified and trained to extract an actual dataset for the plaque characterization process.

Shibutani et al. [18] proposed a deep learning- (DL-) based automated classification method for coronary atherosclerotic plaques. Optical frequency domain imaging (OFDI) provides important features and patterns that are presented in an image.

Tiwari et al. [19] introduced an ensemble framework for the cardiovascular disease prediction process. Machine learning (ML) techniques are also used here to detect the exact cause of disease. A random forest-based classifier is used here to classify the type of disease based on the patient's condition.

Xu et al. [20] proposed a multifeature fusion method for the plaque vulnerability detection process. Region of Interest (ROI) is first identified by the fusion method that provides a feasible set of data for the analysis process. The proposed method is mainly used to determine the risk factor of plaque disease.

Apostolopoulos et al. [21] introduced a deep learning approach to the cardiovascular disease (CVD) detection process. Myocardial perfusion imaging is used here that captures the exact details of CVD. The convolutional neural network (CNN) algorithm is used here for the CVD detection process that finds the important set of features from an image.

Zhang et al. [22] proposed a stacking-based model for the acute myocardial infarction (AMI) process. Select from a model (SFM) is used here to extract the effective set of features presented in an image. A certain set of classifiers are used here to determine the exact class of AMI disease.

Lee et al. [23] introduced an artificial intelligence- (AI-) based method for coronary artery calcium scoring (CACS). The proposed method is also used for the plaque analysis process that produces the necessary data for various processes. The deep learning (DL) approach is used here to discover the details from medical images. DL reduces the classification process's latency rate, enhancing the CACS system's efficiency.

Liu et al. [24] proposed a vulnerable plaque detection method for intravascular optical coherence tomography (IVOCT) images. The main aim of the proposed method is to improve the quality accuracy in the plaque vulnerable detection process. The deep convolutional neural network (DCNN) method is used here to classify the patterns and features presented in medical images.

Wang et al. [25] introduced a multifactor method for the plaque detection process. The proposed method's main aim is to improve the plaque burden increase (PBI) rate. The proposed method finds the exact measurement rate in the plaque detection process.

Zhou et al. [26] proposed a deep belief network- (DBN-) based method for ultrasound image analysis. The proposed method is used to determine the effective features presented in ultrasound images. Contrast-enhanced ultrasonography (CEUS) captures the exact details of patients' internal organs.

### 2.1. Proposed Characteristic Extraction Technique (CET) Using Knowledge Learning (KL)

The proposed technique for ultrasonic image processing with knowledge learning (KL) analysis is designed to expel the errors in manual clinical trials based on smart computing systems and intelligent image processors based on play characteristic extraction. The ultrasonic data or image input processing for updating characteristic extraction obtains an optimal selection of disease features and trained similar datasets. The play characteristics such as personality-induced hyperactivity model, dangerous behavior model, transactional stress moderation model, and constitutional predisposition model are consecutively observed by knowledge learning. Indeed, ultrasonic image input is a routine screening tool for characteristic extraction and diagnosis of cardiovascular disease based on an image processor. However, plaque detected in an ultrasonic image input is considered irrelevant for the diagnosis of cardiovascular disease and thus is marked as false positives (FPs) and is not observed in current ultrasonic data or image screening and processing. Rather than characteristic extraction based on this data analysis, the automated detection of cardiovascular disease based on hard plaque characteristics could take advantage of continuous ultrasonic image screening. It ensures that the disease characteristics and features from image or data processing based on identifying plaque characteristics is the solution for different people affected by cardiovascular disease at different time intervals. The characteristic extraction based on a selection of disease features and trained similar datasets is required from the available disease characteristics relying on image processors. In manual clinical diagnosis, especially cardiovascular disease, diagnosis is considered a critical task involving many features, doctors' decisions, and characteristic extraction. This is usually done by ultrasonic data or image processing based on the output of previous cardiovascular disease-affected patient tests. The play characteristic extraction is used for analyzing disease attributes dependent on the knowledge, experience, and intuition of the doctor; hence, it can affect the service to patients with cardiovascular disease; therefore, in the decision taken by doctors in an automated way, the precision of diagnosis cardiovascular disease has not been significant. This training practice causes false rates and high medical costs. The proposed CET-KL is presented in Figure 1.

In ultrasonic input image processing, the different disease attributes and characteristic extraction of cardiovascular disease detection are analyzed and training of the processing device concurrently through knowledge learning. Therefore, this learning process is responsible for image and data features in a continuous manner with less false rate and time complexity. The segmentation and data extraction are modeled for plaque characteristics with weak knowledge updates that are unidentifiable. The consecutive image analysis is precisely to be employed for the next image processing within the knowledge update and segmentation at different intervals. The image data feature observation and plaque detection outputs in feature mislead problems of reducing false rates and abnormal characteristics of ultrasonic image input analysis, respectively, then

(1) $$\begin{array}{c} UL{\left(i_{m},d_{a}\right)}_{ob}=\underset{ob=T}{\sum }\left[{\left(i_{m}\right)}_{p}-1-\left(\frac{{\left(i_{m}\right)}_{p}}{\sum {\left(i_{m},d_{a}\right)}_{ob}}\right)\right], \end{array}$$

where the variables *i*_*m*_ and *d*_*a*_ are used to represent the ultrasonic image and data observation based on an image processor through knowledge learning. The standard knowledge update for disease characteristics  *Dc*, the maximum ultrasonic data analysis precision based on characteristic extraction *Ch* = 1 achieves high ultrasonic *i*_*m*_ and *d*_*a*_ analysis using the variable processor configuration of disease feature observation. The maximum input image characteristic extraction of *Ch* = 1 achieves high ultrasonic *i*_*m*_ and *d*_*a*_ for the disease analysis of identifying available problems based on the feature or data observation. If *ob* represents the number of ultrasonic images and data observations, (*i*_*m*_)_*p*_ denotes the image processor analysis instance. Instead, *T* is not constant due to smart computing system and intelligent image processors for image and data feature processing as *Ch* ∈ [0, 1] is varying constraints. Therefore, *Ch* = 1 is not detected in any interval  *T*, outputs in false rate, and abnormal characteristics. This problem is referred to as play characteristics, extraction of features, and data based on ultrasonic image input of cardiovascular disease-affected peoples. The assisting knowledge learning is used in this proposed technique for cardiovascular disease detection, analysis with maximum configuration, and precise training of the image processor observation.

### 2.2. Knowledge Learning-Based Characteristic Extraction

In knowledge learning based on characteristic extraction, observation through ultrasonic image, and data input analysis, the patient's characteristics, features, and data can be analyzed and then specific selection disease features and provide training for similar datasets in the image processor through the variable processor configuration. The knowledge base guides the ultrasonic image and data processing performed under KL. The knowledge base consists of plaque characteristic observation to identify the abnormal characteristics and extraction occurrence in cardiovascular disease detection as in Equation (1). The probability of image and data features are segmented in  *T* without abnormal characteristics and false rate, i.e., *ρ*(*f*_*α*_) is given by

(2) $$\begin{array}{c} \rho \left(f_{\alpha }\right)=\frac{\sum_{ob\in T}F_{R}}{\sum_{i\in 1}A_{C}}{Sg}^{\left(i_{m}/p\right).\delta .ob}. \end{array}$$

In Equation (2), the variables *F*_*R*_ and *A*_*C*_ are used to represent the false rate and abnormal characteristic detection in cardiovascular disease detection at different time intervals  *T*. The actual unwanted characteristics and false rates are identified and further processed to reduce this problem. Similarly, the characteristic extraction relies on images, and data features are segmented based on the condition 1 − ((*i*_*m*_)_*p*_/∑(*i*_*m*_, *d*_*a*_)_*ob*_) computed using  *δ*. The first input for maximizing the probability of characteristic extraction based on plaque detection of *Ch* = 1 is the variable processor configuration. This is a cardiovascular disease detection based on ultrasonic image input; therefore, the data extraction is processed depending on the false rate and error detection  *ob* ∈ *T*. The association of disease attributes and acquired data based on *T* instances is used to estimate the output for feature and data segmentation analysis of plaque characteristics. This false rate identification is computed as

(3) $$\begin{array}{c} F_{R}\forall ob\in T=\left[\left(1-\delta \right)\;\frac{i_{m}}{A_{C}}.-Ch.\frac{i_{m}}{T}-\left(A_{C}-F_{\delta }\right)\right],{\left(i_{m}\right)}_{p}\in T. \end{array}$$

In Equation (3), the false rate and error occurrence in cardiovascular disease detection based on the available ultrasonic image and data is analyzed through KL in  *T*. If the condition *F*_*R* ∀ *ob* ∈ *T* computed for data extraction is required, then nonproblematic segmentation is achieved. The abnormal characteristics in the available information maximize *δ*, then defacing the functions to reduce the errors and false rates. In Figure 2, the disease detection and information extraction processes are illustrated.

The extracted characteristics are used for identifying the plaque data and the regions across different  *d*_*o*_. In this process,  *ρ*(*f*_*a*_) is accounted for its maximum  *P*_ext_ such that  *f*_*T*_ is valid. For the  *F*_*R*_ in the segmented region, the correlation is performed such that  *Ch* = 1 or  0 (true or false) is estimated. For the true  *Ch*, the data extraction is performed, whereas for the false  *Ch* condition, detection is performed (refer to Figure 2). The cardiovascular disease detection and analysis holds the available information of image and data features based on the disease characteristics by training image processor; based on the serving ultrasonic image input as  {*Ch*, *F*, *F*_*δ*_, *ρ*(*i*_*m*_)}, post the characteristic extraction with *f*_*α*_ identification in *T* at different time intervals. The detection of abnormal characteristics and errors from data extraction based on *f*_*α*_ and *F*_*R*_∀ *i* ∈ *T* is observed from the knowledge base, and it is updated based on plaque characteristic detection in cardiovascular disease identification. The output is addressed for characteristic extraction and associated with data extraction concurrently analyzed for error occurrence. In this technique, the outcomes are detected using knowledge update, which depends on *F* and  *Ch*. Based on the condition, ∑_*i*∈*ob*_(*i*_*m*_)_*ob*_ = *i*_*m*_ , and *F*_*δ*_ and  *ρ*(*i*_*m*_) are the training input analysis instances as in Equation (1). In this manuscript, let  *f*_*T*_ and  *f*_*δ*_ represent the data extraction input based on ultrasonic image and data analysis for both instances. It refers to the characteristic extraction of image and data observation and plaque extraction outputs with precise outcomes based on analysis precision. Therefore, the plaque extraction (*P*_ext_) is computed as

(4) $$\begin{array}{c} P_{\mathrm{ext}}=\left(\frac{f_{T}*f_{\delta }}{ob}\right), \end{array}$$

where this characteristic extraction analysis observes the cardiovascular disease-affected patients and their symptoms to prevent those associated plaque characteristics based on the data analysis. Therefore, the plaque extraction constraints are substituted in the instance of cardiovascular disease detection and processing using ultrasonic imaging expelled for precise outcomes, respectively.

(5) $$\begin{array}{c} f_{\text{T}}=\underset{i\in ob}{\sum }{\left(i_{m}\right)}_{p}=\left[\frac{Ch\;\sum_{ob\in T}\left({\left(i_{m}\right)}_{ob}/F_{R}\right)}{Ch\sum_{i\in T}A_{C}}\right]. \end{array}$$

Such that,

(6) $$\begin{array}{c} f_{\delta }=\frac{\sum_{i\in ob}\sum_{i\in T}{\left(i_{m}\right)}_{p}-\left(1-{f_{\delta }}_{ob}\right)}{\sum_{i\in ob}\left(f_{T}-f_{\delta }\right)}. \end{array}$$

From Equations (5) and (6), *S*_*ch*_ is computed for precise characteristic extraction based on *i*_*m*_, and *F* with *δ* is to evaluate the reliable outcomes. Instead, the data extraction of *f*_*T*_ relies on *F* and *Ch*, whereas the errors and abnormal characteristics in the computation of cardiovascular disease detection and analysis are based on *f*_*δ*_ and  *i*_*m*_ constraints. The training of the processing device is based on  *f*_*δ*_, and *Ch* results in either 1 or 0 require different characteristic extraction of ultrasonic image, and data observation is analyzed successfully. In this instance of  *P*_ext_ = *f*_*δ*_, then available problems do not occur at the time of cardiovascular disease detection. The data and feature segmentation in Equation (1) does not identify any plaque detection in another process. In this knowledge, the update is performed through training input, and the plaque extraction relies on *Ch* = 1 and *F*_*R*∀ *ob* ∈ *T* = *F*_*R*∀ *i* ∈ *ob* for which the abnormal characteristics and false rates of cardiovascular disease observed in patients are analyzed at different time intervals *T*. The plaque extraction based on the condition 0 < *Ch* < 1 is acute for the weak knowledge updates through *P*_ext_ = ((*f*_*T*_∗*f*_*δ*_)/*ob*) that is observed and analyzed at different time intervals of *P*_ext_(*T*) = *f*_*T*_(*T* − (*A*_*C*_/*F*_*R*_)) + *f*_*δ*_(*T*)∀ *ob* ∈ *T* and  *i* ∈ *T*, respectively. The learning illustration for false identification is portrayed in Figure 3.

The input  *P*_ext_ is first validated for  *Ch* = 1 or  *Ch* = 0 condition. If  *Ch* = 1, then  *T* ∈ *i*_*m*_ is analyzed contrarily, if *Ch* = 0, then  *A*_*c*_ is validated. Based on the  *f*_*δ*_,  *A*_*c*_ ≠ *F*_*R*_, and  *A*_*C*_ = *F*_*R*_ is analyzed. The unmatching output is used for false rate analysis, preventing segment-based detection. The  *A*_*C*_ and  *A*_*C*_ ≠ *F*_*R*_ are alone updated in the  *K*_up_∀ *d*_*o*_ in the further detection process (refer to Figure 3). The plaque detection and false identification through consecutive image analysis for plaque characteristics is the detection of errors and analysis time based on  (*T* − (*A*_*C*_/*F*_*R*_)). It is the feature that misleads at *T* intervals, where  *A*_*C*_ ≠ *F*_*R*_. This first ultrasonic image input analysis is based on *f*_*T*_, and *ρ*(*i*_*m*_) is evaluated through the knowledge update instance *f*_*T*_(*T* − (*A*_*C*_/*F*_*R*_)) based on  *Ch*. This plaque extraction is analyzed with problematic and nonproblematic play characteristic feature extraction through KL for disease characteristics are detected; this knowledge update *K*_up_ is modeled using the processor configuration given as

(7) $$\begin{array}{c} K_{\text{up}}=\frac{\text{C}h*{\left[\rho \left(i_{m}\right)/\left(i_{m}-f_{T}\right)\right]}^{{∁}_{\alpha }}*\left(T-\left(A_{C}/F_{R}\right)\right)}{{\left(i_{m}\right)}_{p}}. \end{array}$$

Equation (7) follows the first outcome of data and feature segmentation based on plaque characteristics; extraction is output in *Ch* = 1 and  *A*_*C*_ = 0, and  *i*_*m*_ = 1. Hence, it is considered as the selection of disease features and trained similar data for characteristic extraction of *K*_up_ = ∑_*i*∈*ob*_(*i*_*m*_)_*p*_ or *d*_*a*_ until this condition  [1 < *T* − (*A*_*C*_/*F*_*R*_) < *T* ] is observed. Therefore, based on the consecutive ultrasonic image analysis in cardiovascular disease, detection based on *i*_*m*_ and *d*_*a*_ is jointly analyzed and processed through KL  [*T* − (*A*_*C*_/*F*_*R*_)]. The previous cardiovascular disease affected patient's characteristics; extraction features and data are compared with current data extraction of  *Ch*, and  *ρ*(*i*_*m*_) is the available information in smart computing systems and intelligent image processors based on the configuration. In particular, the plaque characteristic modification is analyzed based on Equation (1) performed in the segmentation, and data extraction is to increase plaque extraction. The probability of *P*_ex_ depending on the knowledge-based update is competed as

(8) $$\begin{array}{c} \rho \left(P_{\text{ex}}\right)=\left(\frac{\rho \left(i_{m}\cup d_{a}\right)}{\rho \left(A_{C}*F_{R}\right)}\right). \end{array}$$

The data extraction for cardiovascular disease detection using ultrasonic input images and data processing or screening relies on knowledge learning. The characteristic extraction is used to associate training input for updating the knowledge base. The above conditions are validated to the segmentation of image and data features using an image processor. The characteristic changes based on environment and people based on varying patient observations for analyzing cardiovascular disease detection and plaque extraction probabilities at different time intervals of abnormal characteristic information detection with disease attribute analysis. The cardiovascular disease-affected people characteristics are identified and performed to reduce the disease characteristics through knowledge learning. Then, the abnormal characteristics, errors, and false identification were perceived using KL processing. If the condition  *ρ*(*i*_*m*_) > *ρ*(*d*_*a*_), then abnormal characteristic in cardiovascular disease detection, as in Equation (8), is responsible for the optimal selection of disease features based on  *F* and  *Ch*. The characteristic extraction is verified with available information observation through *ob* in cardiovascular disease detection. This consecutive image analysis helps to reduce the extraction ratio in plaque extraction analysis output in strong knowledge updates to maximize plaque characteristic extraction.

## 3. Discussion

This section presents the comparative analysis of the proposed method's performance using the MATLAB experimental analysis. In this analysis, the ultrasonic image inputs from [27] are used for training and validation. This dataset provides 450 patient data for training and 50 for testing with the optimal ejection factor seeded at 45 : 55. The image quality is classified as good for 366 records and poor for 84 records. The metrics precision, characteristic update, training rate, extraction ratio, and time factors are compared for the above inputs. The methods MFFM [20], MS-MT u-net [23], and AAPDF [16] are used in the “Related Works” section for comparison. First, the self-analysis for the considered attributes is presented in this section, followed by the comparative analysis. In Table 1, the features, estimation probability, and the  *Ch* for different segments are tabulated.

For varying segments, the features are extracted based on  *ρ*(*f*_*a*_) such that  *P*_ext_ identifies  *Ch*. If *Ch* is true (1), then  *P*_ext_ is high and hence the features. This has an impact on the varying segments such that  *F*_*R*_∀ *ob* is addressed in preventing fewer  *K*_up_. Depending on the knowledge update, further validations are provided in maximizing the features preventing false rates. Therefore, as the segments vary, the  *Ch*∀ *ρ*(*f*_*a*_) is analyzed in maximizing feature extraction. As the extraction increases, the precision is high.  Table 2 presents the training rate, detection, and knowledge update for the varying *f*_*T*_.

For the varying  *f*_*T*_, the training rate is determined using the identified segments and their corresponding  *K*_up_. Depending on the detection, improvements are performed for which further training is provided. For varying detection rates, the segment-based classification and *P*_ext_ are performed for data and features, preventing false rates. Therefore, the training rate is improved based on segments and updates. The experimental results are tabulated in Tables 3 and 4 for a sample input in this subsection.

### 3.1. Precision

This proposed technique satisfies the high precision for identifying abnormal characteristics and false rates in cardiovascular disease detection (refer to Figure 4). The false rate and errors are mitigated based on the condition for selection of disease features from ultrasonic images and data input processing due to characteristic extraction through knowledge learning. The disease characteristic identification is based on the attributes of the disease using data extraction and image analysis from the previous cardiovascular disease characteristics to the current cardiovascular disease characteristics for identifying false rates. The abnormal characteristics in ultrasonic image processing are based on the configuration instances. The false rates and error identification maximize the characteristic extraction along with updating data; hence, the plaque detection is increased. In the ultrasonic input image and data processing, the image processor is used to extract the characteristics, preventing feature misleads in data extraction. Therefore, the first input image and data are to be observed for the condition  *Ch* ∈ [0, 1]; based on this analysis, precision has to achieve in the segmentation and data extraction for retaining the weak knowledge updates. In the proposed technique, the data extraction is used for updating the knowledge through training input to maximize precision.

### 3.2. Characteristic Update

The characteristic update is high in this proposed technique for cardiovascular disease detection based on plaque detection compared to the other factors in characteristic extraction of specific training of the processing device (refer to Figure 5). In this analysis, the image and data features based on cardiovascular disease are detected at different time intervals. In the condition for increasing plague characteristics in current disease attributes (as in Equation (6)), the processor configuration and data extraction achieved analysis precision in which cardiovascular disease detection is computed. In this proposed technique, play characteristic extraction is determined. The maximum precision for disease characteristic observation and postdisease attributes are analyzed in the segmentation process. This identified false rate maximizes the plaque extraction, continuously preventing abnormal characteristics. From this differing ultrasonic image input, the data extraction is computed to update the training input for the knowledge update represented. In this proposed technique, the training input is based on plaque detection; therefore, the feature and data changes and process segmentation are less false rate.

### 3.3. Training Rate

This proposed technique achieves a high training rate for characteristic extraction and their precision analysis (refer to Figure 6). The time factor, false rate, and errors are mitigated based on features and data analysis for whether abnormal characteristics are identified in cardiovascular disease detection based on problematic or nonproblematic data extraction through knowledge learning. The quality and data extraction help identify the errors and abnormal characteristics in the disease attribute analyzed. Cardiovascular disease detection addresses the abnormal characteristics and false rates with their accuracy and the condition 1 − ((*i*_*m*_)_*p*_/∑(*i*_*m*_, *d*_*a*_)_*ob*_) based on time factor sequence identifying an optimal selection of disease characteristics in cardiovascular disease detection using an update of the knowledge base from the previous characteristic extraction with the current data extraction performing both the instances. Hence, the play characteristic extraction is analyzed to increase the ultrasonic image and data input following differing disease features. In this proposed technique, the defined image and data feature are valid until updating the knowledge to maximize the training rate.

### 3.4. Extraction Ratio

This proposed technique achieves a high extraction ratio in cardiovascular disease detection at different time intervals based on the image and data features used for identifying the false rates (refer to Figure 7). The abnormal characteristic detection and time factor are mitigated through an intelligent image processor for ultrasonic image processing, and fake rate identification depends on analyzing the characteristic extraction through knowledge learning. The information analysis is based on hard plaque characteristics from a knowledge base. The data extraction is used for detecting errors and false rates at different time intervals. The disease attribute analysis is based on segmentation and knowledge update from training input in cardiovascular disease based on the condition ∑_*i*∈*ob*_(*i*_*m*_)_*ob*_ = *i*_*m*_ , and *F*_*δ*_ and  *ρ*(*i*_*m*_) are the training input analysis instances. The plaque characteristics are used to identify the false rate and errors at different time intervals. Similarly, identifying the abnormal features is observed to increase the training rate and address errors based on plaque extraction; hence, the extraction ratio is increased.

### 3.5. Time Factor

This proposed characteristic extraction technique achieves a high time factor for cardiovascular disease detection based on plaque characteristics (refer to Figure 8). The false rate, abnormal characteristic detection, and problems based on *f*_*α*_ and *F*_*R*_∀ *i* ∈ *T* are observed from the knowledge base being updated based on plaque characteristic detection. In cardiovascular disease identification for detecting false rates and problems in disease attributes is due to varying disease characteristics. The image and data feature analysis to increase the variable processor configuration is based on knowledge base information through the learning process. This problem is addressed in segmentation and data extraction from ultrasonic image processing based on the previous characteristic extraction verification in each instance of plaque detection, reducing the false rates through knowledge learning. Therefore, the plaque extraction (*P*_ex_) is computed for improving the characteristic extraction and the selection of disease features at different time intervals. In the proposed technique, abnormal characteristic detection is used for false rate identification and increasing the time factor. Tables 5 and 6 present the comparative analysis results for attributes and segments.

The proposed method maximizes the precision, update, training rate, and extraction ratio by 10.35%, 10.27%, 9.28%, and 11.18%, respectively, whereas it reduces the time factor by 7.6%.

The proposed method maximizes the precision, update, training rate, and extraction ratio by 11.19%, 9.16%, 8.22%, and 11.66%, respectively, whereas it reduces the time factor by 9.38%.

## 4. Conclusion

This article introduced a characteristic extraction technique for improving cardiovascular disease detection using ultrasonic imaging. The proposed approach relies on knowledge learning to enhance the data and image analysis in detecting cardiovascular plaques. The proposed method extracts the data and image features using precise segmentation and data correlation using the image processor. The knowledge base is updated based on the characteristic extraction and disease-related attributes. This update is performed to adapt the image processor configuration in managing different inputs. For further improving the training over distinct features, the extraction possibility is analyzed such that the knowledge base is prevented from unnecessary updates. This further confines the time factor in improving the training rate such that false rates are confined. The segmentation process classifies new attributes and features without increasing the image analysis complexity, maximizing the data extraction. For the varying segments, the proposed method maximizes the precision, update, training rate, and extraction ratio by 11.19%, 9.16%, 8.22%, and 11.66%, respectively, whereas it reduces the time factor by 9.38%.

## Figures and Tables

**Figure 1:** Proposed CET-KL.

**Figure 2:** Disease detection and information extraction.

**Figure 3:** Learning illustration for false rate identification.

**Figure 4:** Precision comparisons.

**Figure 5:** Characteristic update comparisons.

**Figure 6:** Training rate comparisons.

**Figure 7:** Extraction ratio comparisons.

**Figure 8:** Time factor comparisons.

**Table 1:** Features, estimation probability, and *Ch*.

Segments	*ρ*(*f*_*a*_)	*P*_ext_ (%)	*Ch*	Features
1	0.21	46.09	0	1
2	0.28	51.67	0	3
3	0.36	58.36	0	5
4	0.47	65.21	1	10
5	0.52	72.58	1	8
6	0.49	69.21	0	7
7	0.69	80.14	1	12
8	0.81	85.21	1	16
9	0.89	91.57	1	21
10	0.95	93.58	1	26

**Table 2:** Training rate, detection, and knowledge update.

*f*_*T*_	Segments identified	*K*_up_ (%)	Detection	Training rate
100	1	40.39	0.564	0.972
200	5	48.36	0.614	0.962
300	4	45.21	0.589	0.782
400	6	52.14	0.632	0.732
500	7	68.21	0.784	0.787
600	12	78.24	0.921	0.712
700	10	71.25	0.896	0.618
800	14	81.62	0.953	0.64

**Table 3:** Feature extraction and region detection.

Input	Extraction	Identified region
		

**Table 4:** Segmentation and plaque detection.

Identified region	Segmentation	Detection
		

**Table 5:** Comparative analysis for attributes.

Metrics	MFFM	MS-MT u-net	AAPDF	CET-KL
Precision	0.667	0.746	0.818	0.9506
Update (%)	51.44	61.58	69.66	81.439
Training rate	0.693	0.796	0.865	0.9703
Extraction ratio	58.29	72.21	82.45	93.349
Time factor (s)	3.41	2.98	2.41	1.598

**Table 6:** Comparative analysis for segments.

Metrics	MFFM	MS-MT u-net	AAPDF	CET-KL
Precision	0.637	0.722	0.827	0.9524
Update (%)	51.46	63.36	74.54	81.443
Training rate	0.719	0.811	0.867	0.9634
Extraction ratio	58.86	68.23	83.66	93.576
Time factor (s)	3.46	2.96	2.42	1.287

## Data Availability

The data that support the findings of this study are available from the corresponding author upon reasonable request.
